The article "Effects of Glimepiride Combined with Recombinant Human Insulin Injection on Serum IGF-1, VEGF and TRACP-5b Oxidative Stress Levels in Patients with Type 2 Diabetes Mellitus" was published in 2022. Journal: Evid Based Complement Alternat Med.

# Effects of Glimepiride Combined with Recombinant Human Insulin Injection on Serum IGF-1, VEGF and TRACP-5b Oxidative Stress Levels in Patients with Type 2 Diabetes Mellitus

**DOI:** 10.1155/2022/4718087

**Published:** 2022-05-06

**Authors:** Xue Chen, Sheng Kang, Zeqing Bao

**Affiliations:** ^1^Department of Pathology and Pathophysiology, Zhaoqing Medical College, Zhaoqing, Guangdong, China; ^2^Department of Endocrinology, Lanling County People's Hospital, Linyi, Shandong, China; ^3^Department of Basic Medicine, Zhaoqing Medical College, Zhaoqing, Guangdong, China

## Abstract

**Objective:**

This study was designed to explore the effect of glimepiride combined with recombinant human insulin injection on serum insulin-like growth factor 1 (IGF-1), vascular endothelial growth factor (VEGF), tartrate-resistant acid phosphatase 5b (TRACP-5b) and oxidative stress levels in patients with type 2 diabetes.

**Methods:**

A total of 217 patients with type 2 diabetes who were treated in our hospital from November 2018 to March 2020 were selected and divided into control group and treatment group. The control group was treated with glimepiride (*n* = 107). The study group was given glimepiride and recombinant human insulin injection) (*n* = 107). The levels of blood glucose, blood lipids, IGF-1, VEGF, TRACP-5b, and oxidative stress in the two groups were measured, respectively. We summarize the main results as follows. Insulin resistance index (HOMA-IR), fasting blood glucose (FPG), 2h postprandial blood glucose (2hBG), serum glycated hemoglobin (HbA1c), triglyceride (TG), total cholesterol (TC), serum malondialdehyde (MDA), reactive oxygen species (ROS), VEGF, and TRACP-5b levels were significantly lower than those before treatment, and the degree of reduction in the study group was greater than that in the control group (*P* < 0.05). The levels of insulin (INS), insulin beta cell function index (HOMA-beta), superoxide dismutase (SOD), glutathione peroxidase (GSH-Px), and IGF-1 were significantly higher than those before treatment. Further, the study group demonstrated better results than the control group (*P* < 0.05).

**Conclusion:**

Glimepiride combined with recombinant human insulin injection can improve insulin sensitivity, reduce insulin resistance, significantly reduce glucose and lipids in patients, reduce the occurrence of oxidative stress, promote the secretion of oxidative resistance enzymes, lower the vascular endothelial growth factor (VEGF), reduced the formation of new blood vessels, and inhibit the growth and metastasis of cancer cells. Additionally, we found out that glimepiride combined with recombinant human insulin injection had a good prognosis for patients; it significantly reduced the bone resorption marker TRACP-5b and prevented the occurrence of complications such as osteoporosis. The combined use of the two is more effective than glimepiride alone. In conclusion, glimepiride combined with recombinant human insulin injection has higher application value in the treatment of patients with type 2 diabetes.

The article "Effects of Glimepiride Combined with Recombinant Human Insulin Injection on Serum IGF-1, VEGF and TRACP-5b Oxidative Stress Levels in Patients with Type 2 Diabetes Mellitus" was published in 2022. Journal: Evid Based Complement Alternat Med.

## 1. Introduction

Type 2 diabetes is a chronic metabolic disease that mostly occurs after the age of 35 to 40, accounting for more than 90% of diabetic patients [1], with the main feature of hyperglycemia. Long-term hyperglycemia can easily cause lipid metabolism, hemorheology, and oxidative stress and easily induce a series of complications, which seriously affect people's health and life [2]. At present, metformin combined with other hypoglycemic drugs is often used in clinical treatment. However, due to the particularity of the disease, patients need long-term medication. The efficacy of metformin and other hypoglycemic drugs is reduced and there are many adverse reactions, so the treatment effect is not ideal. Recombinant human insulin is a polypeptide hormone [3]. It is synthesized by DNA technology and has 51 amino acid residues in its molecular structure, which is the same as the structure of human insulin produced by human insulin beta cells. This drug is a short-acting insulin preparation [4–6], often used in combination with intermediate- or long-acting insulin preparations [7]. Glimepiride is a long-acting sulfonylurea oral hypoglycemic agent, which can improve insulin resistance and insulin sensitivity by stimulating pancreatic *β* cells to secrete insulin [8, 9]. Both of them have been widely recognized in the treatment of type 2 diabetes. At present, there are few literature studies on the treatment of type 2 diabetes with glimepiride combined with recombinant human insulin injection. Based on the aforementioned observation, our study mainly explored the effects of combined medication on insulin indicators, glucose metabolism indicators, and oxidative stress indicators in patients, so as to provide reference for clinical treatment.

## 2. Materials and Methods

### 2.1. General Information

A total of 217 patients with type 2 diabetes who were treated in our hospital from November 2018 to March 2020 were selected and divided into the control group and study group. The control group was treated with (glimepiride, *n* = 107), while the study group was treated with (glimepiride and recombinant human insulin injection, *n* = 107). There were 64 males and 44 females in the study group; the age ranged from 63 to 74 years, with an average age of (66.37 ± 4.71) years; the disease duration was 2 to 10 years, with an average disease duration of (6.25 ± 1.33) and the mean BMI (24.53 ± 3.27). In the control group, there were 67 males and 40 females; the age ranged from 61 to 73 years, with an average age of (65.84 ± 4.36) years; the disease duration was 2 to 10 years, with an average disease duration of (6.77 ± 1.58) and the mean BMI (23.92 ± 3.18). There was no significant difference in general data between the two groups of patients, and there was no statistical significance (*P* > 0.05), which was comparable. See Table 1.

The article "Effects of Glimepiride Combined with Recombinant Human Insulin Injection on Serum IGF-1, VEGF and TRACP-5b Oxidative Stress Levels in Patients with Type 2 Diabetes Mellitus" was published in 2022. Journal: Evid Based Complement Alternat Med.

### 2.2. Inclusion and Exclusion Criteria

Inclusion criteria for our study were as follows: met the diagnostic criteria for type 2 diabetes: FPG ≥7.0 mmol/L; no other complications; normal cognitive function; and patients and their families informed the study and signed the consent form. On the other hand, exclusion criteria were type 1 diabetes mellitus and gestational diabetes mellitus; autoimmune disease; recent use of insulin coagulation and fibrinolytic drugs; tumor diseases; and allergic to the drugs in this study.

## 3. Methods

The control group was given glimepiride (Shandong Xinhua Pharmaceutical Co., Ltd., Chinese medicine Zhunzi: H20010571), orally 30 minutes before breakfast, the initial dose was 1 mg/time, 1 time/d, and the blood sugar control was stable in the later stage, and the dose was maintained. If the blood sugar control is not ideal, the maximum dose can be increased to 3 mg/time, 1 time/d. The treatment was continued for 3 months. On the basis of treatment, the observation group was additionally given recombinant human insulin injection (United Laboratories International Holdings Co., Ltd., approved by the State Drug Administration: S20100015), and the dosage was usually 0.3–1.0 U per kilogram of body weight per day, with three meals in the morning, noon and evening, The course of treatment was 12 weeks.

### 3.1. Observation Method

Before and after treatment, 5 mL of fasting venous blood was drawn from both groups in the morning, and the supernatant was collected after centrifugation to measure the levels of insulin, glucose metabolism, blood lipids, oxidative stress, insulin-like growth factor 1 (IGF-1), vascular endothelial growth factor (VEGF), and tartrate-resistant acid phosphatase 5b (TRACP-5b). We describe them one by one. (1) Insulin indicators: plasma insulin (INS), insulin *β*-cell function index (HOMA-*β*), insulin resistance index (HOMA-IR), HOMA-*β* = 20 × INS/(FPG-3.5), HOMA-IR = (FPG × FINS)/22.5, and INS was detected by electrochemiluminescence. (2) Glucose metabolism and blood lipid indexes: fasting blood glucose (FPG), 2h postprandial blood glucose (2hBG), serum glycosylated hemoglobin (HbA1c), triglyceride ester (TG), total cholesterol (TC), fasting blood glucose (FPG), and 2h postprandial blood glucose (2hBG) were measured by the glucose oxidase method. Serum glycated hemoglobin (HbA1c) was measured with a PfimusPOQ glycated hemoglobin detector, and blood lipid levels were detected with an automatic blood lipid detector (model: MC-6200) to detect triglyceride (TG) and total cholesterol (TC) levels. (3) Oxidative stress indicators: serum malondialdehyde (MDA), superoxide dismutase (SOD), glutathione peroxidase (GSH-Px), and ROS, the detection method is an enzyme-linked immunosorbent assay kit for detecting MDA, GSH-Px, and ROS was provided by Nanjing Jiancheng Bioengineering Research Institute, and the serum SOD was detected by chemical colorimetry; (4) IGF-1 level: solid-phase, enzyme-labeled chemiluminescence immunoassay, instrument: IMMULITE/IMMUIITE 1000; (5) VEGF level: VEGF was detected by the enzyme-linked immunosorbent assay, and the kit was purchased from Wuhan Boster Bioengineering Co. Ltd., China. (6) Bone specificity was determined using kits provided by IDS Company in the United Kingdom and R&D Company in the United States using tartrate-resistant acid phosphatase-5b (TRACP-5b). All the above tests were conducted by professionals. (7) Comparison of the therapeutic effects of the two groups of patients: According to the relevant provisions in the “Guiding Principles of Clinical Research on New Chinese Medicines” as the evaluation standard, markedly effective: symptoms improved and 2 h PG levels decreased by ≥ 40%; effective: symptoms improved and 2 h PG levels decreased 20% to 39%; invalid: no improvement or even worsening of symptoms. The total effective rate of treatment = marked rate + effective rate.

The article "Effects of Glimepiride Combined with Recombinant Human Insulin Injection on Serum IGF-1, VEGF and TRACP-5b Oxidative Stress Levels in Patients with Type 2 Diabetes Mellitus" was published in 2022. Journal: Evid Based Complement Alternat Med.

### 3.2. Statistical Analysis

SPSS26.0 was used for statistical analysis. The measurement data were represented by the independent sample *t*-test, which was represented by (±*s*), and the count data were represented by the percentage [n (%)], which was represented by the X^2^ test. Pie charts were created using GraphPad Prism8. (*P* < 0.05) was considered statistically significant.

## 4. Results

### 4.1. Comparison of General Data of the Two Groups of Patients

There was no significant difference in general data between the two groups of patients, and there was no statistical significance (*P* > 0.05), see Table 1.

### 4.2. Comparison of Insulin Indexes before and after Treatment between the Two Groups of Patients

Insulin (INS) in the two groups increased after treatment relative to before treatment, and the degree of decrement in the study group was greater than that in the control group (*P* < 0.05). The degree of increment in the study group was significantly greater than that in the control group (*P* < 0.05); the insulin resistance index (HOMA-IR) in both groups after treatment was significantly lower than that before treatment, and the study group was better than the control group after treatment (*P* < 0.05), as shown in Table 2.

### 4.3. Comparison of Glucose Metabolism and Blood Lipid Indexes between the Two Groups before and after Treatment

After treatment, fasting blood glucose (FPG) was lower than before treatment, while the study group was significantly lower (*P* < 0.05); 2 h postprandial blood glucose (2hBG) was significantly lower than before treatment, and the degree of decrease in the study group was better than that in the control group (*P* < 0.05); the levels of serum glycosylated hemoglobin (HbA1c) after treatment were also decreased compared with those before treatment, and the degree of decrease in the research group beat the control group (*P* < 0.05); triglyceride (TG) and total cholesterol (TC) were lower after treatment. Before treatment (*P* < 0.05), the research group was better than the control group, see Table 3.

### 4.4. Comparison of Oxidative Stress Indicators before and after Treatment between the Two Groups of Patients

Serum malondialdehyde (MDA) and ROS in the two groups after treatment were significantly lower than those before treatment (*P* < 0.05). After treatment with superoxide dismutase (SOD) and glutathione peroxidase (GSH-Px), MDA and ROS were significantly higher than before treatment (*P* < 0.05), see Table 4.

### 4.5. Comparison of Serum IGF-1, VEGF, and TRACP-5b between the Two Groups of Patients before and after Treatment

After treatment, IGF-1 in the two groups was significantly higher (*P* < 0.05), while VEGF and TRACP-5b were significantly lower after treatment (*P* < 0.05), as shown in Table 5.

### 4.6. Comparison of the Effective Rate of Treatment between the Two Groups of Patients

We present a comparison of the treatment effective rate between the study group and the control group (98.13% vs 87.85%). The treatment effective rate in the study group was significantly higher than that in the control group (*P* < 0.05). See Table 6 and Figure 1.

## 5. Discussion

The pathogenesis of T2DM is complex. It is generally accepted by the academic community that T2DM is caused by the combined action of genetic factors and environmental factors. Type 2 diabetes is a common endocrine and metabolic disease, and its incidence is on the rise [10]. Type 2 diabetes is a chronic disease with elevated blood sugar mainly due to impaired biological action and/or insufficient secretion of insulin. Long-term high blood sugar can easily lead to abnormal lipid metabolism and hemorheology and cause various complications. Therefore, it is very important to undergo effective treatment in a timely manner. Glimepiride is a long-acting sulfonyl gland hypoglycemic drug with unique dual pharmacological properties. It stimulates the secretion of pancreatic islet cells and at the same time facilitates the release of insulin to achieve rapid hypoglycemic effect and helps glucose metabolism outside the pancreas [11, 12]. Glimemil has the characteristics of fast binding to receptors, short time of interaction with membrane receptors, and fast hypoglycemia [13]. It can also increase nonoxidative metabolism by increasing glucose transporters, thereby reducing blood sugar [14, 15]. The results of this study showed that the post-treatment insulin resistance index (HOMA-IR), fasting blood glucose (FPG), 2 h postprandial blood glucose (2hBG), serum glycated hemoglobin (HbA1c), triglyceride (TG) in the study group and control group, total cholesterol (TC), serum malondialdehyde (MDA), ROS, VEGF, and TRACP-5b levels were significantly lower than those before treatment, and the degree of reduction in the study group was greater than that in the control group, glimepiride may improve insulin sensitivity, reduces insulin resistance, and has always reduced blood glucose and blood lipids in patients. The reduction in blood glucose inhibited the inflammatory infiltration of neutrophils and reduced the occurrence of a large number of oxidative intermediates. Therefore, serum malondialdehyde (MDA) and ROS were reduced. The oxidative stress response is greatly reduced, and the secretion of antioxidant enzymes is promoted, including superoxide dismutase (SOD) and glutathione peroxidase (GSH-Px), which further reduces the occurrence of oxidative stress and inhibits the disease. A meta-analysis of data from 11 included RCTs conducted by Morvaridzadeh revealed no support convincing evidence as to a significant increasing effect of pomegranate intake in TAC (SMD: 0.43; 95 %CI: −0.19, 1.06), Gpx (SMD: 0.18, 95% CI: −0.25, 0.62, *p* = 0.4) and paraxonase (SMD: 0.36, 95% CI: −0.50, 1.22, *p* = 0.41) as well as not significant decrease in malondialdehyde (MDA) (SMD: −0.81, 95% CI: −1.79, 0.09, *P* = 0.08) [16]. The levels of insulin (INS), insulin beta cell function index (HOMA-beta), superoxide dismutase (SOD), glutathione peroxidase (GSH-Px), and IGF-1 were significantly higher than those before treatment, and the research group was significantly higher than the control group. Recombinant human insulin injection was injected into the body, which rapidly increased the insulin content in the body [17]. Insulin *β*-cell function index (HOMA-*β*) were elevated [18] because glimepiride decomposes a large number of free fatty acids in the patient's body, inhibits excessive carbon monoxide synthase, reduces cell damage, and gradually restores islet *β*-cell function normal, so that liver-derived glucose is broken down rapidly, reducing blood sugar in type 2 diabetes patients. The results of this study show that the combination of glimepiride and recombinant human insulin injection increases insulin levels, and insulin can upregulate the expression of vascular endothelial growth factor (IGF-1), so that IGF-1 increases synchronously, which is highly consistent with the results of Younossi's study. Similar to [19], IGF-1 has the functions of lowering blood sugar, lowering blood lipids, relaxing blood vessels, promoting bone anabolism, and maintaining the normal structure and function of bone [20]. The increase of IGF-1 inhibits the occurrence of bone resorption, The bone resorption marker TRACP-5b was significantly reduced, preventing osteoporosis in patients with type 2 diabetes. Previous studies have shown that VEGF is highly expressed in liver cancer and plays an important role in the formation of new blood vessels and tumor growth and metastasis in liver cancer. In this study, VEGF decreased, indicating that the combined use of glimepiride and recombinant human insulin injection can reduce blood sugar and inhibit the inhibition of VEGF in the liver. There is an abnormally high expression of a variety of factors within the tumor, which thereby reduces the occurrence of tumor cells [21]. The effective rate of treatment in the study group was significantly higher than that in the control group (*P* < 0.05).

The article "Effects of Glimepiride Combined with Recombinant Human Insulin Injection on Serum IGF-1, VEGF and TRACP-5b Oxidative Stress Levels in Patients with Type 2 Diabetes Mellitus" was published in 2022. Journal: Evid Based Complement Alternat Med.

The combined use of glimepiride and recombinant human insulin injection can effectively exert its synergistic effect, which is beneficial to improve the metabolic defects of the patient's body, so as to control the glucose and lipid metabolism of the patient within the normal range and reduce the occurrence of oxidative stress [22], reduces vascular endothelial growth factor (VEGF), and reduces the formation of new blood vessels. Further, the combined use inhibits the growth and metastasis of cancer cells, has a good prognosis for patients, and significantly reduces the bone resorption marker TRACP-5b. In addition, the combined use of glimepiride and recombinant human insulin injection prevents the occurrence of complications such as osteoporosis. The combined use of the two is more effective than glimepiride alone. In conclusion, glimepiride combined with recombinant human insulin injection has a higher application value in the treatment of patients with type 2 diabetes.

The article "Effects of Glimepiride Combined with Recombinant Human Insulin Injection on Serum IGF-1, VEGF and TRACP-5b Oxidative Stress Levels in Patients with Type 2 Diabetes Mellitus" was published in 2022. Journal: Evid Based Complement Alternat Med.

## Figures and Tables

**Figure 1:** Comparison of the effective rates of treatment in the two groups of patients.

**Table 1:** Comparison of general data of the two groups of patients.

	Study group (*n* = 107)	Control group (*n* = 107)	*t/x* ^2^	*P*
Gender (male/female)	64/44	67/40	0.255	0.614
Age	63∼74	61∼73		
Mean age	66.37 ± 4.71	65.84 ± 4.36	0.854	0.394
Course of disease	2∼10	2∼10		
Mean course	6.25 ± 1.33	6.77 ± 1.58	2.604	0.01
Mean BMI	24.53 ± 3.27	23.92 ± 3.18	1.383	0.168

**Table 2:** Comparison of insulin indexes before and after treatment in two groups of patients ($\bar{x}$ ± *s*).

Groups	N	INS (mmol/L)		HOMA-*β*		HOMA-IR	
		Before treatment	After treatment	Before treatment	After treatment	Before treatment	After treatment
Study group	107	11.53 ± 2.34	18.78 ± 3.92	38.56 ± 0.23	160.20 ± 13.67	4.56 ± 0.37	2.23 ± 0.36
Control group	107	11.27 ± 3.02	15.41 ± 3.72	38.23 ± 0.26	67.69 ± 7.53	4.59 ± 0.40	3.52 ± 0.47
*t*		0.704	6.451	1.278	61.315	0.57	22.539
*P*		0.482	<0.001	0.208	<0.001	0.569	<0.001

**Table 3:** Comparison of glucose metabolism and blood lipid indexes between the two groups of patients before and after treatment ($\bar{x}$ ± *s*).

Groups	n	FPG (mmol/L)		2 hPG (mmol/L)		HbA1c (%)		TC (mmol/L)		TG (mmol/L)	
		Before treatment	After treatment	Before treatment	After treatment	Before treatment	After treatment	Before treatment	After treatment	Before treatment	After treatment
Study group	107	9.48 ± 1.34	5.47 ± 0.56	13.24 ± 1.92	7.61 ± 1.39	9.77 ± 1.23	7.05 ± 0.63	5.72 ± 1.09	4.12 ± 1.12	2.87 ± 0.66	2.11 ± 0.97
Control group	107	9.50 ± 1.38	8.04 ± 0.73	13.47 ± 2.07	10.29 ± 1.64	9.65 ± 1.21	8.12 ± 1.29	5.77 ± 1.12	5.34 ± 1.57	2.84 ± 0.62	2.68 ± 1.14
*t*		0.108	28.894	0.843	12.895	0.719	7.71	0.156	6.544	0.343	3.939
*P*		0.914	<0.001	0.4	<0.001	0.473	<0.001	0.427	<0.001	0.732	<0.001

**Table 4:** Comparison of oxidative stress indexes before and after treatment in two groups of patients ($\bar{x}$ ± *s*).

Groups	n	MDA (mmol/L)		SOD (U/L)		GSH-px (mol/L)		ROS (IU/mL)	
		Before treatment	After treatment	Before treatment	After treatment	Before treatment	After treatment	Before treatment	After treatment
Study group	107	5.91 ± 0.63	2.66 ± 0.39	64.71 ± 4.27	97.31 ± 18.21	24.37 ± 4.57	29.03 ± 3.94	644.49 ± 32.84	573.87 ± 14.83
Control group	107	5.89 ± 0.57	4.24 ± 0.52	64.59 ± 3.86	84.23 ± 13.16	24.53 ± 5.39	26.35 ± 5.57	645.31 ± 33.57	614.51 ± 27.36
*t*		0.244	25.144	0.216	6.022	0.234	4.063	0.181	13.508
*P*		0.807	<0.001	0.829	<0.001	0.815	<0.001	0.857	<0.001

**Table 5:** Comparison of serum IGF-1, VEGF, and TRACP-5b between the two groups of patients before and after treatment ($\bar{x}$ ± *s*).

Groups	n	IGF-1 (ng/mL)		VEGF (mmol/L)		TRACP-5b (U/L)	
		Before treatment	After treatment	Before treatment	After treatment	Before treatment	After treatment
Study group	107	43.51 ± 9.08	73.68 ± 9.57	130.21 ± 26.37	95.72 ± 13.64	10.61 ± 1.39	4.63 ± 0.07
Control group	107	43.17 ± 9.07	62.45 ± 8.34	129.44 ± 25.95	104.30 ± 15.74	10.29 ± 1.64	4.72 ± 0.03
*t*		0.161	9.151	0.215	4.261	1.54	12.224
*P*		0.872	<0.001	0.83	<0.001	0.125	<0.001

The article "Effects of Glimepiride Combined with Recombinant Human Insulin Injection on Serum IGF-1, VEGF and TRACP-5b Oxidative Stress Levels in Patients with Type 2 Diabetes Mellitus" was published in 2022. Journal: Evid Based Complement Alternat Med.

**Table 6:** Comparison of the effective rate of treatment between the two groups of patients ($\bar{x}$ ± *s*).

Groups	n	Markedly effective	Effective	Ineffective	Total
Study group	107	72	33	2	98.13
Control group	107	40	54	13	87.85
X^2^					8.675
*P*					0.003

## Data Availability

The datasets used and analyzed during the current study are available from the corresponding author on reasonable request.
